# Astrocyte Elevated Gene-1 Mediates Glycolysis and Tumorigenesis in Colorectal Carcinoma Cells *via* AMPK Signaling

**DOI:** 10.1155/2014/287381

**Published:** 2014-04-16

**Authors:** Hong-tao Song, Yu Qin, Guo-dong Yao, Zhen-nan Tian, Song-bin Fu, Jing-shu Geng

**Affiliations:** ^1^Department of Pathology, The Affiliated Tumor Hospital of Harbin Medical University, Harbin 150040, China; ^2^Department of Medical Genetics, Harbin Medical University, Harbin 150086, China

## Abstract

To investigate the role of AEG-1 in glycolysis and tumorigenesis, we construct myc-AEG-1 expression vector and demonstrate a novel mechanism that AEG-1 may increase the activity of AMPK by Thr172 phosphorylation. The higher expression levels of AEG-1 in colorectal carcinoma cells were found but showed significant difference in different cell lines. To study the role of AEG-1 in colorectal cells, myc-AEG-1 vector was constructed and transfected into NCM460 colonic epithelial cells. We observed consistent increasing of glucose consumption and lactate production, typical features of anaerobic glycolysis, suggesting that AEG-1 may promote anaerobic glycolysis. Moreover, we noted that AMPK phosphorylation at Thr172 as well as pPFK2 (Ser466) was increased in NCM460 cells overexpressing AEG-1. Compound C may block AMPK and PFK2 phosphorylation in both control and AEG-1-overexpressed cells and decrease the glucose consumption and lactate production. The present findings indicated that reduced AEG-1 protein levels by RNAi may decrease the glucose consumption and lactate production in HCT116 colorectal carcinoma cells. The present identified AEG-1/AMPK/PFK2 glycolysis cascade may be essential to cell proliferation and tumor growth. The present results may provide us with a mechanistic insight into novel targets controlled by AEG-1, and the components in the AEG-1/AMPK/PFK2 glycolysis process may be targeted for the clinical treatment of cancer.

## 1. Introduction

The tumorigenesis of cancer cells involves numerous genetic and epigenetic lesions, resulting in the critical alteration of multiple cellular restraints. Many oncogenes may induce persistent activation of unusual cell procedures and promote carcinoma growth [1, 2]. It is widely accepted that tumor cells shift their metabolism away from respiration toward anaerobic glycolysis, to achieve excessive cell growth, proliferation, and resistance to apoptosis [3]. Most tumor cells exhibit increased glycolysis and take this metabolic pathway as a main source of their energy supply to generate ATP. This is the so-called Warburg effect [4]. Thus, the increasing of glycolysis of tumor cells may be recognized as an important event in tumorigenesis and potential target for antitumorigenesis for cancer therapy. Nowadays, tremendous progress has been made in understanding of the molecular mechanisms of tumorigenesis, especially in the signaling corresponded for its increased glycolysis, such as PI3K-AKT-mTOR signaling [5, 6]. However, it is still largely unknown for the complicated network of increasing glycolysis of tumorigenesis.

Astrocyte elevated gene-1 (AEG-1) is originally cloned as a gene induced in primary human fetal astrocytes (PHFA) infected with HIV-1 or treated with tumor necrosis factor-*α* (TNF-*α*). It is also revealed that AEG-1 was significantly elevated in subsets of breast carcinoma, melanoma, and malignant glioma cell lines compared to their normal cell counterparts. The correlation of AEG-1 with many carcinomas affords the potential that AEG-1 plays a crucial role in the oncogenic transformation and tumorigenesis [7, 8]. Previous study showed that AEG-1 expression was markedly induced by Ha-ras, which was transcriptionally mediated through the PI3K signaling pathway [9, 10]. Other reports revealed AEG-1 functions in cell transformation, which is an important event in tumorigenesis [11–13]. It was also demonstrated that AEG-1-expressing tumors have increased microvessel density throughout the entire tumor sections, which also contributes to the tumorigenesis [14].* In vitro* angiogenesis studies further reveal that AEG-1 promotes tube formation in Matrigel and increases invasion of human umbilical vein endothelial cells with increased expression of angiogenesis markers, such as hypoxia-inducible factor 1-*α* (HIF-1*α*) [7, 9, 15, 16]. It is noted that AEG-1 may increase the expression of HIF-1*α*, which is a critical factor for glycolysis [17, 18]. Besides HIF-1*α*, AEG-1 is also proved to activate AMPK, which may also be of potential to promote glycolysis and tumorigenesis [8, 13, 19]. AMP-activated protein kinase (AMPK) is a highly conserved heterotrimeric kinase complex and activated under conditions of energy stress. The phosphorylation of the activation loop threonine is absolutely required for AMPK activation [20, 21]. It is found that AEG-1 reduces the ATP/AMP ratio and activates AMP kinase, which induces AMPK-dependent autophagy [13, 22, 23]. Interestingly, AEG-1-induced autophagy by AMPK protects cells from apoptosis, which might benefit tumor cells for surviving under pharmacological conditions [19].

Although AEG-1 exhibits several regulatory functions in tumorigenesis, it is intriguing whether there are other aspects of tumorigenesis regulated by AEG-1 and how AEG-1 activates intracellular signaling pathways. In the present study, we showed that AEG-1 may upregulate glycolysis in NCM460 human colonic epithelial cells by activation of AMPK signaling. The activated AMPK then phosphorylates 6-phosphofructo-2-kinase (PFK-2) and induces the synthesis of fructose 2,6-bisphosphate, which is a key intermediate product of glycolysis. Moreover, inhibition of AMPK activity in NCM460 cells or interfering AEG-1 expression in HCT116 human colon carcinoma cells reversed the increased glycolysis. All these results will help to understand a novel clue regarding the role of AEG-1 as a potential cancer therapeutic in tumor cells, as well as the molecular mechanism of tumorigenesis.

## 2. Materials and Methods

### 2.1. Chemicals and Materials

Dulbecco's modified Eagle's medium (DMEM), trypsin, and fetal bovine serum (FBS) were obtained from Hyclone (Hyclone, Logan, Utah) and M3 media from Sigma (St. Louis, MO, USA). The anti-AEG-1 antibody was from Epitomics (San Diego, CA, USA). Anti-beta-actin was purchased from Millipore (Billerica, MA, USA). pAMPK (T172) and AMP-activated protein kinase (AMPK) antibody were from Cell Signaling Technology (Beverly, MA, USA), while pPFK2 (S466) and phosphofructokinase-2 (PFK2) were from Santa Cruz (Santa Cruz, California, USA). Myc antibody was from Thermo Scientific (MA, USA). The AMPK inhibitor Compound C was provided by MERCK (Billerica, MA, USA). Other reagents used were of reagent grade or higher.

### 2.2. Assays of Cell Culture

NCM460 cell line was a nontransfected human colonic epithelial cell line, while HCT116 cell line was established from a primary colon carcinoma and widely used in the colon cancer research. The NCM460 cells were introduced from INCELL Corporation (San Antonio, TX, USA) and HCT116, HT29, and SK/S cells from the American Type Culture Collection (Manassas, VA, USA). NCM460 cells were cultured in M3 media and HCT116 in DMEM with 10% fetal bovine serum (FBS) and 1% antibiotics at 37°C in a 95% air/5% CO_2_ atmosphere at constant humidity. Following, transfection was carried out when the cell confluent was 80–90% using Lipofectamine 2000, and cell was harvested at 48 h after transfection with lysis buffer (PBS+1% Triton + proteinase inhibitors). All the transfection manipulations, including AEG-1 overexpression and siRNA, were performed as transient transfection, not stable clones. For Compound C treatment, 20 *μ*M Compound C was applied to cells and lasted for 2 h to block AMPK activity.

### 2.3. Vectors Construction

The myc-AEG-1 construct for overexpression of AEG-1 in NCM460 cells was generated by subcloning the PCR-amplified human AEG-1 coding sequence into pRK5-myc vectors. To reduce the endogenous AEG-1 protein level in HCT116 cells, we generated another AEG-1 RNAi pSuper vector with the following oligonucleotides, 1# AACAGAAGAAGAAGAACCGGA and 2# GAAATCAA AGTCAGATGCTA (Invitrogen) as previous report [24]. All these generated vectors were sequenced.

### 2.4. Assay of Western Blot

Western blot was performed as standard procedures. To extract proteins, cultured cells were sonicated with lysis buffer (PBS) with 1% Triton X-100 and proteinase inhibitors. The protein concentration of each extract was measured by the BCA Protein Assay kit (Thermo Scientific Pierce, Rockford, IL, USA). Equal amounts of the proteins from each extract were loaded into and separated by SDS-PAGE. The proteins were transferred onto PVDF membranes following standard procedures. The membranes were then blocked by 5% nonfat dry milk in TBST (TBS with 0.1% Tween 20, pH 7.6) for 1 h at room temperature and probed overnight by proper primary antibodies diluted in TBST at 4°C. After 3 times of washing with Tris-buffered saline and Tween (TBST) at room temperature for 10 min each, the membranes were incubated with proper secondary antibodies diluted in TBST (1 : 10,000 for both goat anti-rabbit and goat anti-mouse IgG) for 1 h at room temperature. After another 3 times of membrane washing with TBST at RT for 10 minutes each, proteins were detected by Pierce ECL Western blotting substrate kit (Thermo Scientific/Pierce, Rockford, IL, USA) reagent and exposed to film (Kodak).

### 2.5. RNA Extraction and Real-Time PCR Assay

Total RNAs were extracted from cells using Trizol reagent (Invitrogen, Carlsbad, CA, USA). RNA was subjected to reverse transcription with reverse transcriptase as manufacturer's instructions (Fermentas Inc., Hanover, MD, USA). Quantitative real-time PCR was performed using the Bio-Rad iQ5 system using Bio-Rad proprietary iQ5 software (Hercules, CA, USA), and the relative gene expression was normalized to internal control as beta-actin. Primer sequences for SYBR Green probes of target genes were as follows: AEG-1: TTGAAGTGGCTGAGGGTGAA and TACGCTGCTGTCGTTTCTCT and beta-actin: GAGACCTTCAACACCCCAGC and ATGTCACGCACGATTTCCC.

### 2.6. Measurements of Glucose and Lactate

Glucose consumption and lactate production were performed as the following step. A total of 6–8 × 10^4^ cells per well were seeded in 12-well plates for 24 h and then treated with or without Compound C for 48 h. Cell numbers were counted before measurements using a hemocytometer. The medium was collected and the glucose and lactate levels are analyzed. Glucose was measured spectrophotometrically using an Olympus AU5400 (Olympus Corporation, Tokyo, Japan). The lactate was measured using a RXL MAX system (Dade Behring, Deerfield, IL, USA). The glucose consumption and lactate production were normalized to cell numbers.

### 2.7. Statistical Analysis

All results of western blots, real-time PCR, and biochemical assays across time were presented as mean ± SEM. from three independent experiments at least. Data from western blots were analyzed by ImageJ software.* P* values were calculated using Student's *t*-test for normally distributed data, and the values 0.05 (∗), 0.01 (∗∗), and 0.001 (∗∗∗) were assumed as the levels of significance for the statistic tests carried out.

## 3. Results

### 3.1. AEG-1 Was Highly Expressed in Human Colon Carcinoma Cells

Numerous reports have revealed the essential role of AEG-1 in the development and progression of cancer. Aberrant elevation of AEG-1 expression frequently occurs in human cancers, including breast cancer, glioma, melanoma, esophageal squamous cell carcinoma, prostate cancer, hepatocellular carcinoma, and gastric cancer. Moreover, AEG-1 is found to be differentially overexpressed in adenoma and cancer cells, whereas it is weakly expressed in normal mucosa [8, 25, 26]. Although AEG-1 is potentially correlated with colorectal carcinomas, it is not well understood how AEG-1 performs in colorectal carcinomas. Thus, the mRNA and protein levels of AEG-1 in colorectal carcinomas were investigated in canonical human colon carcinoma cell lines, such as HCT116, HT29, and S/KS. The protein levels of AEG-1 in HCT116, HT29, and S/KS cells were significantly increased than that of NCM460 cells, by 16.2-, 13.4-, and 15.9-fold (Figures 1(a) and 1(b)). Results of real-time PCR analysis also showed that the transcriptional level of AEG-1 was extremely high in these three colorectal carcinoma cells, increased by 18.7-, 20.1-, and 22.3-fold in HCT116, HT29, and S/KS cells compared to that of NCM460 (Figure 1(c)). The extremely high transcription of AEG-1 affords its protein translation in colorectal carcinoma cells, which contributes to the tumorigenesis transcriptional homeostasis impairment from many aspects.

### 3.2. AEG-1 Promoted Anaerobic Glycolysis* via* AMPK in NCM460 Human Colonic Epithelial Cells

To study the role of AEG-1 in colon cancers, we next generate and validate the myc-tagged AEG-1 overexpression vectors and transfect it into NCM460 human colonic epithelial cells to elevate aberrant AEG-1 gene expression. After transfection, the NCM460 cells were harvested for subsequent western blot, to confirm the overexpression of myc-AEG-1. The myc blots indicated that human-derived AEG-1 was expressed in NCM460 cells (Figure 2(a)). Performing metabolic assays of glucose consumption and lactate production in AEG-1-overexpressed NCM460 cells, the present results indicate that glucose consumption and lactate production in AEG-1-overexpressed cells increased by 4.6- and 4.8-fold compared with those in nontransfected control cells, respectively, and the values show significant differences (Figures 2(b) and 2(c)). This consistent increasing of glucose consumption and lactate production is a typical feature of anaerobic glycolysis and suggests that AEG-1 may promote anaerobic glycolysis. It has been reported that AEG-1 may cause a significant increase of AMPK phosphorylation at Thr172 [13]. While the phospho-AMPK (Thr172) may activate AMPK activity and phosphorylate 6-phosphofructo-2-kinase at Ser466 sites, which may induce the synthesis of fructose 2,6-bisphosphate, a potent stimulator of glycolysis. Therefore, we assume that AEG-1 upregulates anaerobic glycolysis by increasing AMPK/PFK2 axis. To test this, we take biochemical assays to investigate the phosphorylation level of both AMPK and PFK2. We find that AMPK phosphorylation at Thr172 is increased in NCM460 cells overexpressed of AEG-1 (Figure 2(d)). However, the total level of AMPK showed no significant change. For AMPK may promote glycolysis by phosphorylating PFK2, we next check the PFK2 phosphorylation at Ser466 in NCM460 cells with AEG-1 overexpression. Similarly, the pPFK2 (Ser466) also increases in AEG-1-overexpressed cells (Figure 2(d)). All the present findings suggest that AEG-1 might activate anaerobic glycolysis* via* AMPK signaling.

### 3.3. Inhibition of AMPK Signaling Reverses AEG-1-Mediated Increasing of Glycolysis

We have described that AEG-1 may increase the phosphorylation of AMPK and PFK2 and promote anaerobic glycolysis. To confirm these findings, we design to inhibit AMPK activity and test whether this will reduce PFK2 phosphorylation and anaerobic glycolysis under AEG-1-overexpressed conditions. The activity of AMPK could be inhibited by Compound C. It is shown that Compound C may antagonize AICAR (AMPK activator) by blocking the uptake of AICAR into cells [27]. Although AEG-1 activates AMPK phosphorylation, Compound C could block AMPK phosphorylation in both control and AEG-1-overexpressed NCM460 cells. PFK2 also showed similar results and AEG-1 may not activate PFK2 phosphorylation in the presence of Compound C (Figure 3(a)). Then, we examined the anaerobic glycolysis in both AEG-1-overexpressed and nontransfected cells. As expectedly, Compound C drastically reduced AEG-1-induced glucose consumption and lactate production by ~38.7% in AEG-1 nontransfected cells. Moreover, Compound C could further decrease the glucose consumption and lactate production by ~48.2% and ~49.4% compared to AEG-1-transfected cells (Figure 3(b)). Thus, these findings confirmed that AEG-1 may promote anaerobic glycolysis by AMPK-PFK2 axis, and inhibition of AMPK may reverse AEG-1-mediated increasing glycolysis.

### 3.4. Downregulation of AEG-1 Expression Reverses AEG-1-Mediated Increasing of Glycolysis in HCT116 Tumor Cells

It was shown that AEG-1 was highly expressed in human colon carcinoma cells and enhanced anaerobic glycolysis* via* AMPK in NCM460 cells. We proposed that ectopic expression of AEG-1 in colon carcinoma cells was responsible for the activated anaerobic glycolysis. To test this hypothesis, we constructed AEG-1 RNAi pSuper vectors to decrease the endogenous AEG-1 expression in HCT116—a widely used human colon carcinoma cell line. Then, we examined the AEG-1 protein levels and found that the AEG-1 expression was decreased in these transfected cells than that of controls (Figure 4(a)). Next, we examined the glucose consumption and lactate production and found that they were inhibited by AEG-1 RNAi (Figure 4(b)). Moreover, our results suggested that decreased AEG-1 protein levels may inhibit cell migrations in HCT116 cells. This result confirmed that blocking energy production by AEG-1 RNAi indeed impaired tumor metastasis (Figure 4(c)). Based on the above results, these findings support the notion that AEG-1 may be critical for anaerobic glycolysis in colon carcinoma cells, and the inhibition of AEG-1 expression may restore the ectopic anaerobic glycolysis in these tumor cells.

## 4. Discussion

Astrocyte elevated gene-1 (AEG-1) expression increases in multiple cancers and plays a crucial role in oncogenic transformation and angiogenesis, which are essential components in tumor cell development, growth, and progression to metastasis. Moreover, AEG-1 directly contributes to resistance to chemotherapeutic drugs, another important hallmark of aggressive cancers [8, 12]. Multitissue northern blots containing total RNA of normal human organs revealed that AEG-1 mRNA is ubiquitously expressed at varying levels in all organs [28]. Expression analysis in cell lines revealed that AEG-1 expression is significantly higher in breast, prostate, esophageal, and liver cancer and melanoma, malignant glioma, and neuroblastoma cell lines in comparison to their normal counterparts [11, 14, 28–31]. These studies provide important insights and a unique perspective on this multifunctional oncogene, AEG-1. However, how AEG-1 enhances tumorigenesis is not well understood. In the present study, we demonstrated a novel mechanism that AEG-1 might increase the anaerobic glycolysis through the activation of AMPK signaling. And inhibition of AMPK activity or downregulation of AEG-1 expression may reverse the effects of AEG-1 on glycolysis (Figure 4(d)).

Anaerobic glycolysis is a metabolic process in which glucose, a sugar molecule, is broken down without the use of oxygen. The phenomenon of anaerobic glycolysis increasing in cancer cells is first described by Otto Warburg (1930) over 70 years ago. Many cells ranging from microbes to lymphocytes use aerobic glycolysis during rapid proliferation, suggesting that it may play a fundamental role in supporting cell growth [4]. Results showed that malignant cells exhibit significantly elevated glycolytic activity even in the presence of sufficient oxygen and consider this phenomenon as the most fundamental metabolic alteration in malignant transformation, or “the origin of cancer cells” [4, 32]. Although the cause-effect relationship between the increase in anaerobic glycolysis and the development of cancer is controversial, increased glycolysis has been consistently observed in many cancer cells of various tissue origins. Indeed, the positron emission tomography (PET) widely used in clinical diagnosis of cancer is based on the fact that cancer cells are highly glycolytic and actively uptake glucose [33, 34]. The Warburg effect can be viewed as a prominent biochemical symptom of cancer cells that reflects a fundamental change in their energy metabolic activity. Several mechanisms have been suggested to affect energy metabolism and thus contribute to the Warburg effect. These mechanisms include (1) mitochondrial defects, (2) adaptation to hypoxic environment in cancer tissues, (3) oncogenic signals, and (4) abnormal expression of certain metabolic enzymes [32].

It seems that malignant cells become additive to glycolysis and dependent on this pathway to generate ATP. Because ATP generation* via* glycolysis is far less efficient (two ATP per glucose) than through oxidative phosphorylation (36 ATP per glucose), cancer cells consume far more glucose than normal cells to maintain sufficient ATP supply for their active metabolism and proliferation [35, 36]. This metabolic feature has led to the hypothesis that inhibition of glycolysis may severely abolish ATP generation in cancer cells and thus may preferentially kill the malignant cells [4]. Recent studies have provided supporting evidence that inhibition of glycolysis may exert preferential effect on cells with compromised mitochondrial function due either to genetic defects or a lack of oxygen [37, 38]. During periods of intracellular metabolic stress, a reduced cellular energy (ATP) level is sensed by AMPK (5′-AMP-activated protein kinase). Previous reports showed that AEG-1 induces noncanonical autophagy involving an increase in expression of ATG5. AEG-1 decreases the ATP/AMP ratio, resulting in diminished cellular metabolism and activation of AMP kinase, which induces AMPK/mammalian target of rapamycin-dependent autophagy [13]. In the present study, our findings reveal that AEG-1 activates anaerobic glycolysis* via* AMPK signaling. This might be helpful for the deep understanding of tumorigenesis. Our work shows that inhibition of AEG-1-AMPK axis by pharmacological treatment (such as Compound C) may be of potential for the clinical biotherapy of tumorigenesis.

## 5. Conclusion

In summary, we identified AEG-1/AMPK/PFK2 signaling for anaerobic glycolysis in human colon carcinoma cells. It is speculated that the frequent hyperactivation of AEG-1/AMPK signaling in the course of the multistep oncogenesis may contribute to the development of the Warburg effect present in many human cancers. Our work may provide a mechanistic insight into novel targets controlled by AEG-1, and the components in AEG-1/AMPK/PFK2 signaling in glycolysis may be targeted for the treatment of cancer.

## Figures and Tables

**Figure 1:** AEG-1 was highly expressed in human colon carcinoma cells. ((a)-(b)) Western blots and histograms showing that AEG-1 protein levels were dramatically increased in HCT116, HT29, and S/KS cells than that in NCM460 cells. Results were averages of four independent experiments. Data represent mean ± SEM. ***P < 0.001. (c) Real-time PCR results showing that AEG-1 mRNA levels were upregulated in HCT116, HT29, and S/KS cells than that in NCM460 cells. Results were averages of four independent experiments. Data represent mean ± SEM. ***P < 0.001.

**Figure 2:** AEG-1 promoted anaerobic glycolysis* via* AMPK in NCM460 human colonic epithelial cells. (a) Western blots showing the overexpression of myc-AEG-1 proteins in NCM460 cells. ((b)-(c)) Biochemical assays showing the increasing of glucose consumptions (b) and lactate productions (c) in AEG-1-overexpressed NCM460 cells, in contrast to controls. Results were averages of four independent experiments. Data represent mean ± SEM. **P < 0.01. (d) Western blots showing that AMPK phosphorylation and PFK2 phosphorylation were increased in AEG-1 overexpressed NCM460 cells. It is noted that the total AMPK or PFK2 protein levels were not altered by AEG-1 overexpression.

**Figure 3:** Inhibition of AMPK signaling reverses AEG-1-mediated increasing of glycolysis. (a) Western blots showing that inhibition of AMPK activity by Compound C (20 *μ*M, 2 h) reduced AMPK phosphorylation and PFK2 phosphorylation in both AEG-1-overexpressed and nontransfected NCM460 cells. (b) Biochemical assays showing that inhibition of AMPK activity ameliorated AEG-1-induced glucose consumption and lactate production in NCM460 cells. Results were averages of four independent experiments. Data represent mean ± SEM. *P < 0.05, **P < 0.01.

**Figure 4:** Downregulation of AEG-1 expression reverses AEG-1-mediated increasing of glycolysis in HCT116 tumor cells. (a) Western blots showing that decreasing AEG-1 protein levels by RNAi reduced AMPK phosphorylation and PFK2 phosphorylation in HCT116 tumor cells. (b) Biochemical assays showing that decreasing AEG-1 protein levels by RNAi reduced glucose consumption and lactate production in HCT116 cells. Results were averages of four independent experiments. Data represent mean ± SEM. **P < 0.01. (c) Images showing that the decreased AEG-1 protein levels may inhibit cell migrations in HCT116 cells. (d) Schematic representation highlighting the molecular link between AEG-1 and glycolysis. AEG-1 may increase the activity of AMPK by Thr172 phosphorylation. The activated AMPK then raises PFK2 activity and promotes glycolysis, as is called Warburg effect.
